# Development and Application of One Separation-Free Safety Tube on the Disposable Infusion Needle

**DOI:** 10.1155/2020/6896517

**Published:** 2020-05-16

**Authors:** Weifen Lu, Qianli Pan, Yinxin Zhou, Wenyu Chen, Hongyan Zhang, Weibo Qi

**Affiliations:** ^1^Department of Respiration, First Hospital of Jiaxing (Affiliated Hospital of Jiaxing University), 314000 Jiaxing, China; ^2^Department of Cardiothoracic Surgery, First Hospital of Jiaxing (Affiliated Hospital of Jiaxing University), 314000 Jiaxing, China

## Abstract

**Objective:**

To develop a new type infusion set and apply it to the clinic, as well as explore its effectiveness in the prevention from needle stick injuries.

**Methods:**

A total of 200 inpatients who were in need of intravenous infusion with a disposable infusion needle were included and randomly divided into two groups: intervention group and control group. Disposable infusion needles with a separation-free safety tube were used in the intervention group, whereas conventional ones were used in the control group. Then, effects of the two types of infusion sets were observed and compared.

**Results:**

As for the operation time for infusion, it was (82.19 ± 1.80) seconds in the intervention group and (83.02 ± 1.83) seconds in the control group, with the difference statistically significant (*P* < 0.05). Besides, the exposure time of the needles after infusion in the intervention group was (3.36 ± 0.17) seconds while (18.85 ± 1.18) seconds in the control group; the difference between which was statistically significant (*P* < 0.05). In terms of the time for needle disposal, (18.60 ± 0.84) seconds was required in the intervention group, while for the control group, it took (18.85 ± 1.18) seconds, and the difference between two groups was of statistical significance as well (*P* < 0.05). Nevertheless, there was no statistically significant difference in the accidental slip rate of the needles as that turned out 0% in both groups (*P* > 0.05). It was worth noting that the block rate of the disposed needles in the intervention group was 100%.

**Conclusion:**

The separation-free safety tube on the disposable infusion needle could instantly block the sharp needle after infusion, which reduces the needle exposure time and lowers the risk of needle stick injuries. In the meantime, the safety tube is convenient to use, and its application can shorten the time for infusion and needle disposal, consequently improving the working efficiency of nurses. As the new type safety tube has above advantages and would not raise the risk of needle slippage, it is worthy of clinical promotion.

## 1. Introduction

According to the World Health Organization (WHO) [1], about 2,000,000 medical staffs suffer from infectious diseases caused by needle stick injuries (NSIs) each year, including hepatitis B virus (HBV), hepatitis C virus (HCV), and human immunodeficiency virus (HIV) [2]. Nowadays, NSIs have become the most serious occupational risk for medical staff. Our hospital is the First Hospital of Jiaxing affiliated to Jiaxing University which is the largest general hospital in Jiaxing city. In our hospital, we have over 2,200 staffs, among which 682 are doctors and 1,061 are nurses. Additionally, each year, there are more than 300 new resident doctors who have received normalization training and over 300 medical students for clinical practice. Statistically, a total of 123 cases of NSIs happened in our hospital in 2018, including 57 cases that occurred in nurses accounting for 46.3%. The main medical sharp instrument responsible for NSIs turned out the intravenous infusion needles (41 cases) which accounted the highest as 33.3%. Among the 41 cases, 2 cases happened during punctuation, 2 cases occurred before reset after needle accidental slippage, 14 cases happened during the process of needle withdrawal, 9 cases happened on the way to the disposal room while the rest 14 cases occurred in the disposal room during needle processing. In order to reduce the incidence of NSIs caused by infusion needles, in this project, we developed a new type safety tube that could not only protect the needle before infusion but also instantly block it after infusion. Details are as follows.

## 2. Subject and Methods

### 2.1. Research Set

The conventional disposable infusion set originally has a protective cover on the needle, which prevents the package and the operator from being punctured and stabbed, and is usually discarded during normal operation. In this project, we transformed such protective cover into a new type one named safety tube. As shown in Figure 1, the inner diameter of the safety tube is slightly larger than the outside diameter of the needle body, and the length of the tube is slightly longer than the total length of the needle head plus the needle body. There is a slit along the length from the front to the middle of the tube. The open end (front) of the tube linked with the slit is in the shape of a “V,” the end of the slit at the middle of the tube is linked with a rectangular hole, and the joint is in the shape of an inverted “V.” The safety tube is in register with the needle, and the fin of the needle is out of the rectangular hole. During infusion, the fin is pushed to make the needle slide along the slit out of the tube, and after infusion, the needle slides back into the tube for safety. The safety tube has been commissioned to a qualified manufacturer and applied to the clinical trial. Meanwhile, it was approved by the hospital ethics committee.

### 2.2. Subject

200 inpatients who were in need of infusion therapy from October to December 2018 were enrolled and randomly divided into the intervention group and the control group. There was no significant difference in age and disease diagnosis between the two groups (*P* > 0.05). In the study, we used disposable infusion needles with a new type separation-free safety tube for the patients in the intervention group and conventional ones with a self-contained protective cover in the control group. Patients in both groups volunteered to participate and had signed informed consent.

### 2.3. Operation Methods

Six ward nurses with proficiency in the conventional infusion operation were selected, including 2 nurses working for 1-3 years, 2 for 3-5 years, and 2 for over 5 years. Before the project, all of them were trained in the operation of this new type safety tube and qualified. In the control group, conventional disposable infusion needles were used. After breathing, the self-contained protective cover was discarded, and the needle was fixed after acupuncture, then separated from the infusion set into a sharps box at the end. Patients in the intervention group were treated with new disposable infusion sets. The specific operation steps were as follows: (1) Instead of being removed after breathing, the safety tube slid to the flexible tube when the fin of the needle was pushed along the slit to make the needle out of the tube. Then, the infusion operation was as the same as the control group. (2) After infusion, the needle was removed. The upper end of the flexible tube away from the needle was raised, and the needle side was lowered to make the safety tube slide down to the needle side. Then, the fin was pushed to slide along the slit into the rectangular hole. The needle was thus blocked, and the whole infusion set was disposed into a special collection bag.

### 2.4. Observation Indicators

(1) Infusion operation time: from the beginning of the breathing to the end of needle fixation after application. (2) Needle exposure time: from the time of needle withdrawal to the time of needle blocked. The latter refers to the time for needle blocked by the safety tube in the intervention group and for needle blocked in a sharps box in the control group. (3) Needle disposal time: from the time of needle withdrawal to the time of needle disposed, wherein the latter refers to the time for needle collection in a special collection bag in the intervention group and in a sharps box in the control group. (4) Accidental slip rate of the infusion needle: the percentage of the cases with accidental needle slippage in the total infusion cases. (5) Needle block rate in the intervention group after disposal: the percentage of the successfully blocked needles (premarked in certain color) in the total amount of needles.

### 2.5. Statistical Methods

The data were input by the statistician and analyzed using the SPSS 21.0 software. The measurement data were presented in the form of mean ± standard deviation (M ± SD). The enumeration data were expressed by frequency and percentage, and the ranked data were determined using the Mann-Whitney *U* of the nonparametric test. *P* < 0.05 was considered statistically significant.

## 3. Results

### 3.1. Infusion Operation Time

As shown in Table 1, the operation time in the intervention group was shorter than that in the control group, with a statistically significant difference (*P* < 0.05).

### 3.2. Needle Exposure Time

As shown in Table 2, the needle exposure time in the intervention group was significantly shorter than that in the control group, with a statistically significant difference (*P* < 0.05).

### 3.3. Needle Disposal Time

As shown in Table 3, the time for needle disposal after infusion in the intervention group was shorter than that in the control group, with a statistically significant difference (*P* < 0.05).

### 3.4. Others

The accidental slip rate of the infusion needles in the intervention group and the control group were both 0%, with no statistically significant difference (*P* > 0.05). In addition, 100 needles in the intervention group were all blocked after disposal with the block rate of 100%.

## 4. Discussion

According to the Centers for Disease Control and Prevention (CDC) statistics [3], 80%-90% healthy medical staffs with infectious diseases are caused by NSIs, of which 80% are nurses. In recent years, as the NSIs happen more often, it has been highly focused in medicine at home and abroad. Various protective measures thus have been studied, such as the development of nursing equipment with safe and protective sets and the application of needle-free products, which have made the incidence of NSIs reduced by 43% [4]. However, due to the high cost of such products, they have not been widely promoted in China at present. Disposable infusion needle is still the main infusion set used in most hospitals, and nurses still have to face the exposed needles with blood and body fluids of patients every day. In addition, nurses need to hold the needles by hand to the disposal room for needle separation after infusion completed. During this process, NSIs could easily happen in either the operators or other people. Among the 41 cases of NSIs in our hospital in 2018, 9 cases happened on the way to find a sharps box. The exposure time of the needle is positively related to the risk of NSIs. Therefore, shortening the needle exposure time is the key to reduce the risk of NSIs. The effective way is to place the sharps boxes in a place where nurses can conveniently reach, such as the bed end or the treatment cart configurated with a sharps box in each ward, which could allow nurses to dispose the used needles in time so as to reduce the exposure time. However, due to the factors like the national conditions, risk of sharps loss, and economic cost, this approach has not been implemented. In most hospitals in China, only the disposal room and the treatment cart in the nursing station are configurated with sharps boxes. From the results of this study, the needle exposure time in the intervention group was significantly shorter than that in the control group (*P* < 0.01). The main reason might be that in the intervention group, the safety tube could slide to the flexible tube when acupuncture and instantly slide back to the needle side after infusion completed, making the needle blocked in time with no necessity searching for a sharps box. The application of the safety tube greatly shortened the needle exposure time, thereby reducing the risk of NSIs. Besides, during the process of needle disposal, the needle should be separated from the infusion set using tools, with the needle placed in a sharps box and the infusion set in a special collection bag. Such treatment is apt to cause NSIs, and 14 cases among the total stick injury cases in our hospital in 2018 just happened during the disposal process. In this study, the blocked needles were disposed in a special collection bag together with the infusion set in the intervention group. Moreover, the needle block rate reached 100% before collection in 10-24 hours, suggesting that the separation-free type safety tube could effectively work, and the sharps box for separation could be no longer needed, which further lowered the incidence of NSIs.

As a large number of infusion operations have to be completed every day, nurses would spend much working time on it. From the data of this group, the infusion operation time of the intervention group was less than that of the control group, and the difference was statistically significant (*P* < 0.01). The main reason can be concluded as the difference in the handling methods for the safety tube in the intervention group and the protective cover in the control group. Moreover, the safety tube is convenient to operate and nurses can grasp it easily. For the protective cover in the control group, it should be removed from the needle and discarded into a waste pail. While for the safety tube in the intervention group, it only needs to slide to the flexible tube when acupunctured, which shortens the operation time. In addition, the needle disposal time after infusion in the intervention group was shorter than that in the control group, with a statistically significant difference (*P* < 0.01). The main reason is that in the control group, the needle should be separated from the infusion set into a sharps box after withdrawal for waste disposal. While in the intervention group, the needle is instantly blocked by the safety tube and placed into the nearest special collection bag. There is no need to process separation; thus, the needle disposal time is reduced. It can be seen that the application of the separation-free safety tube can improve the working efficiency of nurses. In the meantime, the subjects in our study gave no bad feedback and no accidental slippage occurred, indicating that the new type infusion needle is safe to be applied.

The self-contained protective cover of the conventional infusion needle will be discarded routinely before infusion. In this study, the protective cover that should have been discarded was modified into a safety tube, which is with no need for discard and could be used to protect the needle before and after the infusion. It is environmentally friendly. Meanwhile, there was no need for the needles to be separated when disposed in the intervention group, and the use of the sharps boxes therefore could be reduced.

Nowadays, nursing service needs nurses to pay high but repays low income. Moreover, nurses have to face the danger of being infected by NSIs every day, which brings great physical and mental stress. A disposable infusion needle with a separation-free safety tube that can prevent from NSIs is a safe intravenous infusion set available at the present stage. At present, the product has been successfully transferred through the Zhejiang Patent Transfer Platform and is worthy of clinical promotion.

## Figures and Tables

**Figure 1:** Pictures of the normal infusion set and the new type infusion set.

**Table 1:** Infusion operation time (seconds).

Operation time	Median	Interquartile range	*Z*	*P*
Intervention group	82.19	1.69	-3.441	0.001
Control group	82.53	1.27		

**Table 2:** Needle exposure time (seconds).

Exposure time	Median	Interquartile range	*Z*	*P*
Intervention group	3.36	0.16	-12.219	<0.001
Control group	18.52	1.24		

**Table 3:** Needle disposal time (seconds).

Disposal time	Median	Interquartile range	*Z*	*P*
Intervention group	18.39	1.03	-2.151	0.031
Control group	18.52	1.24		

## Data Availability

The data used to support the findings of this study are available from the corresponding author upon request.
